The article "Prevalence of Metabolic Syndrome in Iranian Professional Drivers: Results from a Population Based Study of 12,138 Men" was published in 2012. Journal: PLoS One.

# Prevalence of Metabolic Syndrome in Iranian Professional Drivers: Results from a Population Based Study of 12,138 Men

**DOI:** 10.1371/journal.pone.0031790

**Published:** 2012-02-22

**Authors:** Iraj Mohebbi, Soheil Saadat, Mohammadreza Aghassi, Mahsa Shekari, Maghsuod Matinkhah, Shadi Sehat

**Affiliations:** 1 Occupational Medicine Center, Urmia University of Medical Sciences, Urmia, Iran; 2 Sina Trauma Research Center, Sina hospital, Medical Sciences/University of Tehran, Tehran, Iran; 3 Departement of Endocrinology, Urmia University of Medical Sciences, Urmia, Iran; Howard University, United States of America

## Abstract

**Background:**

It is evident that professional driving is associated with substantial changes in lifestyle habits. Professional drivers are prone to metabolic syndrome (MetS) and its complications because their working environment is characterized by numerous stress factors such as lack of physical activity due to working in a fixed position, disruption in diet, and irregular sleep habits. The aim of the present study was to estimate the prevalence of MetS among long distance drivers residing in West Azerbaijan province in Iran.

**Materials:**

To assess the prevalence of metabolic syndrome among professional long distance drivers, 12138 participants were enrolled in this cross sectional study. The MetS was defined using International Diabetes Federation criteria.

**Results:**

Among12138 participants, 3697 subjects found to be MetS. The crude and age-adjusted rates of MetS were 30.5% and 32.4% respectively. Based on Body mass index (BMI), 5027 subjects (41.4%) were overweight (BMI ≥25.01–30 kg/m2), and 2592 (21.3%) were obese (BMI ≥30.01 kg/m2). The presence of central obesity was more common than other components. The associations of MetS with BMI, pack-year smoking, age, weekly driving duration and driving experiences were significant in the logistic regression. By increasing BMI, pack-year smoking, age, weekly driving duration and driving experiences, odds ratio of MetS was increased.

**Conclusion:**

The study suggests that MetS has become a noteworthy health problem among Iranian long distance drivers. This might be due to the following facts: sitting in a fixed position for long hours while working, cigarette smoking, job stress, unhealthy diet and lack of physical activity. Educational programs should be established for promoting healthy lifestyle and also for early detection and appropriate interventions

## Introduction

A global transition in the disease pattern has been observed, where the relative impact of infectious diseases is decreasing while chronic diseases like cardiovascular disease (CVD) and diabetes are increasingly dominating the disease pattern [1]. In the United States, age-adjusted MetS prevalence among adults population was estimated to be 24–25%. Similarly, the prevalence of MetS in 7 European countries was approximately 23%. It was estimated that 20%–25% of South Asians have developed MetS [2], [3]. In Iran, a high prevalence of this disorder has been documented among general population. According to a nationwide study, the age-standardized prevalence of the metabolic syndrome in Iranian men population was about 28.8% based on the Adult Treatment Panel-III (ATP III) criteria, and 27.5% (95% CI 25.7–29.3) based on the International Diabetes Federation (IDF) definition [4]. In the Tehran study, the age-standardized prevalence of this syndrome in 4397 Iranian men population was estimated 24% and 21% based on the ATP III and the IDF definitions respectively [5], [6]. In Zanjan province in Iran, where the main ethnic groups are Azeries (Turks) and Kurds, the prevalence of this syndrome in men is reported to be 23.1%, based on ATP III criteria [7]. Individuals with MetS have a higher probability of developing diabetes and/or CVD, depending on the number of components present [8]–[12]. It has also been shown that the prevalence of the MetS become more frequent as obesity increases [13], [14]. Central obesity, one of the components of MetS, predicts the occurrence of diabetes and overall cardiovascular risk [9]. It is essential to initiate early detection of these chronic diseases in high risk population groups, so that preventative action can minimize the consequences. In this context, the aim of this study was to estimate the prevalence among Iranian long distance drivers, because they have unusual life styles and their working environment is characterized by numerous stress factors such as lack of physical activity due to working in a fixed position, disruption in diet, and irregular sleep habits [15], [16].

The article "Prevalence of Metabolic Syndrome in Iranian Professional Drivers: Results from a Population Based Study of 12,138 Men" was published in 2012. Journal: PLoS One.

## Results

A total of 12138 male long distance drivers participated in the study. The mean age of the subjects was 37.8 (SD = 10.1) years, ranging from 20 to 67. Considering smoking habits, 8289 (68.3%) of participants were current smokers, 3516 (29.0%) non-smoker, and 333(2.7%) were ex-smokers. The crude and age-standardized prevalence of the MetS were 30.5% and 32.4%. A linear association was observed between age group and prevalence of MetS (Test for trend P-Value <0.001).General characteristics of MetS versus non MetS study subjects are presented in Table 1. The prevalence of individual components of MetS based on age group is reported in Table 2. The central obesity was more common than the other components of MetS (table 2). The number of components of MetS cases (with at least 3 components) increased by increasing age groups (Table 3), and the difference was statistically significant (P Value<0.001). There was a direct association with the BMI and prevalence of MetS (table 4), and the association was statistically significant (P<0.001). Association of MetS with some risk factors was examined by logistic regression. Binary logistic regression was used to examine the relationship between MetS and BMI, smoking, age, weekly driving duration and driving experiences. Based on Hosmer and Lemeshow's goodness of fit test, the model has adequate fit. According to the smoking history participants were divided into 4 groups of non-smokers, 10 pack-years or less, 10.1 to 20 pack-years and more than 20 pack-years smoking. Based on driving experiences they were divided into 3 groups of 10 years or less, 11–20 years and more than 20 years. Mean of weekly driving duration at last year were divided into 3 groups of less than 45 hours, 45 to less than 60 hours and 60 hours or more. BMI categories were divided into 3 groups of 25 or less, 25.1 to less than 30 and 30 or more. Age categories were defined as drivers aged lower than 35, drivers aged 35–49, and drivers aged 50 or more. The results of logistic regression are presented in Table 5. As shown in Table 5, the associations of MetS with BMI, pack-year smoking, age, weekly driving duration in fixed sitting position and history of driving experiences were significant in the logistic regression. BMI and smoking were the variables most significantly associated with the occurrence of MetS. In over weight drivers (BMI = 25.01–30 kg/m^2^) odds ratio of MetS was 6.8 (95% CI; 6.0 to 7.7) compared with their colleagues with normal weight; and also it was 9.4 (95% CI; 8.48 to 10.5) for obese drivers (BMI = More than 30 kg/m^2^). Odds ratio of MetS was 1.2(95% CI; 1.09 to 1.3) for smoking 10 pack-years or less, 2.1(95% CI; 1.8 to 2.5) for smoking 10.1–20 pack-years and 3.5(95% CI; 2.8 to 4.4) in those with smoking more than 20 pack-years in comparison with non-smoker subjects.

**Table 1:** Basic characteristics of MetS versus non MetS subjects.

Characteristic	MetS		P value
	PresentMean(±SD)	AbsentMean(±SD)	
Age (years)	41.3(10.1)	36.2(9.7)	P<0.001
Weekly driving duration(hours)	51.9(20.1)	49.5(20.9)	P<0.001
Driving experiences (years)	14.0(8.9)	10.2(8.0)	P<0.001
Smoking (pack-years)	3.2(8.7)	2.6(7.0)	P<0.001
Waist circumference (centimeter)	102.7(8.0)	88.8(10.8)	P<0.001
Systolic blood pressure (mm Hg)	132.2(15.4)	121.4(12.8)	P<0.001
Diastolic blood pressure (mm Hg)	83.7(10.3)	75.7(9.5)	P<0.001
FBG (mg/dl)	98.8(26.8)	88.2(15.5)	P<0.001
TG (mg/dl)	249.3(134.0)	142.8(95.4)	P<0.001
HDL-C (mg/dl)	40.4(9.0)	45.8(9.3)	P<0.001
BMI(kg/m2)	29.7(3.5)	25.3(3.7)	P<0.001

The article "Prevalence of Metabolic Syndrome in Iranian Professional Drivers: Results from a Population Based Study of 12,138 Men" was published in 2012. Journal: PLoS One.

**Table 2:** Prevalence of the metabolic syndrome and its components according to age groups of study subjects.

	Age groups (years)										All age groups	
Components of MetS	20–24N (%)	25–29N (%)	30–34N (%)	35–39N (%)	40–44N (%)	45–49N (%)	50–54N (%)	55–59N (%)	60–64N (%)	65–69N (%)	Crude prevalence (%)	Age standardized prevalence (%)
Mets	92 (13.5)	440 (17.9)	546 (24.1)	626 (32.6)	554 (34.5)	598 (42.6)	466 (45.7)	253 (46.9)	90 (49.2)	32 (51.6)	30.5	32.4
High Blood pressure	186 (27.4)	666 (27.1)	720 (31.8)	704 (36.6)	668 (41.5)	711 (50.6)	610 (59.9)	383 (71.1)	137 (74.9)	49 (79.0)	39.8	44.6
High triglycerides	200 (29.5)	929 (37.8)	1038 (45.9)	984 (51.2)	849 (52.8)	775 (55.2)	540 (53.0)	254 (47.1)	87 (47.5)	25 (40.3)	46.8	45.5
Low HDL- C	237 (34.9)	880 (35.8)	796 (35.2)	698 (36.3)	515 (32.0)	442 (31.5)	315 (30.9)	161 (29.9)	45 (24.6)	15 (24.2)	33.8	32.7
HighFBG	30 (4.4)	138 (5.6)	204 (9.0)	279 (14.5)	291 (18.1)	391 (27.8)	273 (26.8)	165 (30.6)	64 (35.0)	21 (33.9)	15.3	17.5
Increased Waist circumference	162 (23.9)	821 (33.4)	1038 (45.9)	1033 (53.7)	950 (59.1)	886 (63.1)	686 (67.3)	376 (69.8)	125 (68.3)	47 (75.8)	50.5	51.9

**Table 3:** Number of criteria indicating MetS in study subjects according to age groups.

	Age group (Years)										All age groups	
Number of criteria	20–24	25–29	30–34	35–39	40–44	45–49	50–54	55–59	60–64	65–69	Crude prevalence	Age-adjusted prevalence (%)
0 N (%)	220 (32.4)	694 (28.2)	454 (20.1)	296 (15.4)	205 (12.7)	156 (11.1)	96 (9.4)	33 (6.1)	6 (3.3)	3 (4.8)	2163 (17.8)	16.8
1 N (%)	224 (33.0)	717 (29.2)	619 (27.4)	466 (24.2)	368 (22.9)	251 (17.9)	161 (15.8)	87 (16.1)	37 (20.2)	12 (19.4)	2942 (24.2)	23.9
2 N (%)	132 (19.4)	561 (22.8)	595 (26.3)	488 (25.4)	443 (27.5)	356 (25.3)	262 (25.7)	154 (28.6)	41 (22.4)	14 (22.6)	3046 (25.1)	24.5
3 N (%)	85 (12.5)	353 (14.4)	420 (18.6)	458 (23.8)	382 (23.8)	374 (26.6)	296 (29.0)	143 (26.5)	63 (34.4)	16 (25.8)	2590 (21.3)	22.1
4 N (%)	18 (2.7)	124 (5.0)	148 (6.5)	193 (10.0)	178 (11.1)	220 (15.7)	169 (16.6)	95 (17.6)	30 (16.4)	16 (25.8)	1191 (9.8)	10.9
5 N (%)	0 (.0)	8 (.3)	27 (1.2)	22 (1.1)	32 (2.0)	48 (3.4)	35 (3.4)	27 (5.0)	6 (3.3)	1 (1.6)	206 (1.7)	1.9

**Table 4:** The association of BMI with prevalence of MetS*.

	MetS		
BMI(kg/m^2^)	PresentN (%)	AbsentN (%)	SumN (%)
≤20.0	10 (2.2)	455 (97.8)	465 (100.0)
20.1–25.0	250 (6.2)	3804 (93.8)	4054 (100.0)
25.1–30.0	1787 (35.5)	3240 (64.5)	5027 (100.0)
30.1–35.0	1412 (62.8)	835 (37.2)	2247 (100.0)
>35.1	238 (69.0)	107 (31.0)	345 (100.0)
Total	3697 (30.5)	8441 (69.5)	12138 (100.0)

*P<0.001.

**Table 5:** Odds Ratio (OR) and 95% Confidence Interval (CI) for MetS with some risk factors by using logistic regression.

Variable		B	S.E.	P- value	OR (95% CI)
Weekly driving duration	Less than 45 hours			<0.001	
	60 or more than 60 hours	0.420	0.052	<0.001	1.5(1.4–1.7)
Driving experiences	less than 10 years			0.002	
	20 or more than 20 years	0.249	0.075	0.001	1.3(1.1–1.5)
Smoking	Non Smoking			<0.001	
	10 pack-years or less	0.188	0.054	0.001	1.2(1.1–1.3)
	10.1–20 pack-years	0.753	0.091	<0.001	2.1(1.8–2.5)
	More than 20 pack-years	1.251	0.113	<0.001	3.5(2.8–4.4)
Age	Less than 25 years			<0.001	
	35–49 years	0.296	0.064	<0.001	1.3(1.2–1.5)
	50 or more than 50 years	0.579	0.083	<0.001	1.8 (1.5–2.1)
BMI	25 or less than 25 kg/m^2^			<0.001	
	25.01–30 kg/m^2^	1.915	0.063	<0.001	6.8 (6.0–7.7)
	More than 30 kg/m^2^	2.242	0.054	<0.001	9.4 (8.48–10.5)

The article "Prevalence of Metabolic Syndrome in Iranian Professional Drivers: Results from a Population Based Study of 12,138 Men" was published in 2012. Journal: PLoS One.

## Discussion

The results of the present study demonstrate a noteworthy high prevalence of MetS in drivers. This prevalence is higher than the same age, and sex group in the general population. In a national study, the age-standardized prevalence of the MetS in Iranian men population was about 28.8% based on the ATP III criteria, and 27.5% based on the IDF definition [4]. In the Tehran study, the age-standardized prevalence of this syndrome in 4397 Iranian men population was estimated 24% and 21% based on the ATP III and the IDF definitions respectively [6]. Accordingly, based on ATP III criteria, the prevalence of this syndrome was more than IDF definition in the Iranian population. The above studies overestimate the prevalence of MetS based on ATP III criteria in the Iranian population. It should be noted that the main ethnic groups of our study are the same as those of Zanjan study [7]. In comparison with the Zanjan study, our finding revealed that the rate of MetS was at least 9% more than the general population. Therefore, it seems that the excess prevalence in our survey could be attributed to occupation and life style of our study sample.

A few studies have investigated MetS or its related components in professional long distance drivers. In a cross sectional study, among 429 bus and truck drivers in the central part of Iran, 35.9% of the participants suffered metabolic syndrome based on ATP III criteria [17]. An investigation among bus drivers in Taipei showed that the rates of risk factors for ischemic heart disease among the drivers were significantly higher than comparable groups of skilled workers [18]. In a comparative study done in Norway on cardiovascular risk factors among bus drivers and industrial workers, it was found that bus drivers had higher mean values of serum cholesterol, serum triglycerides, systolic, and diastolic blood pressure [19].

The article "Prevalence of Metabolic Syndrome in Iranian Professional Drivers: Results from a Population Based Study of 12,138 Men" was published in 2012. Journal: PLoS One.

Researchers looked at heart disease in bus drivers from the 1950s. Morris et al. found that rates of coronary heart disease in bus conductors were lower than in less occupationally active bus drivers. This seminal U.K investigation was undertaken using data from two cohorts of British workers [20]. MetS increases the risk for cardiovascular events [21]. On applying modified IDF, we found that the majority of the subjects had at least one abnormal risk factor for MetS. Each component of MetS is a known risk factor for the development of diabetes and CAD. People with MetS are 3–10 times more likely to develop CVD equal with a high risk of morbidity and mortality [2], [22]. Therefore, the excess prevalence of MetS in long distance drivers is a public health concern.

The reasons for excess risk of MetS in professional drivers need to be studied. Some probable explanations are as follows. Many drivers work longer than 45 hours per week. They also work complicated shift systems due to irregular working hours, which lead to inadequate opportunities for recovery and unwinding. [16]. Unhealthy diet and physical inactivity are common in long distance drivers. In adults, high carbohydrate meal consumption is related to hyperinsulinaemia, postprandial hyperglycaemia, and hypertriglycemia that are well known to predict an increase of body fat in working individuals [23], [24]. In Iran, most of inter-city restaurants use high saturated fat for daily cooking. The common meals served in these restaurants are poor in fiber, rich in animal proteins (beef, sheep, veal), and are high in glycemic index (rice, white bread). As shown in table 4, the increase in the BMI was accompanied by a parallel increase in the prevalence of MetS. This may indicate the role of unhealthy diet and physical inactivity in developing MetS in long distance drivers.

Working environment of drivers may also play a role in developing MetS. There are reports indicating that despite regular exercise and a proper diet, subjects under prolonged stress developed metabolic alterations including distinctive central obesity, biochemical changes and a slight hypertension towards the MetS [25]. There is a dose-response relation between exposure to work stressors and risk of the metabolic syndrome, independent of other relevant risk factors [26]. It has been demonstrated that the length of work hours has been a significant factor for both waist circumference and BMI increases in professional drivers and other workers [27], [28]. As shown in Table 5, the odds ratio of Mets was increased with increasing driving time per week. Also odds ratio of MetS in smoker drivers was increased in a statistically significant manner in relation to increasing pack-years of smoking. The odds ratio of the MetS was 1.21(1.09–1.34) for smoking 10 pack-years or less, 2.12(1.78–2.54) for smoking 10.1–20 pack-years and 3.49(2.80–4.36) in those with smoking more than 20 pack-years. There is some evidence that smokers are at greater risk than nonsmokers of becoming MetS [29]–[30]. Based on Lee et al, the relative risk of developing MetS in subjects who smoked more than 20 pack-years was 1.9 (95% CI 1.1–3.7) [31].

The article "Prevalence of Metabolic Syndrome in Iranian Professional Drivers: Results from a Population Based Study of 12,138 Men" was published in 2012. Journal: PLoS One.

This study has several limitations. One of which is the cross-sectional nature of the data, so providing causal inferences of MetS was impossible. The study included men exclusively. Moreover, we did not have a control group of general population to quantify the attributable risk of driving for MetS. We did not examine dietary habits and daily exercise with objective methods, so we were not able to study the exact mechanisms of developing MetS in the study population. Of course, professional driving is associated with substantial changes in lifestyle habits. Physical inactivity is common in long distance drivers. In addition, in the interview with some subjects, we informed the drivers that while they consumed low daily vegetables and little fruit, their foods contained high saturated fat, were rich in animal proteins, and high in glycemic index. The study suggests that MetS has become a noteworthy health problem among the Iranian long distance drivers. This might be due to their working condition which has to be performed in a fix sitting position, job stress, unhealthy diet and physical inactivity. Educational programs should be established for promoting healthy lifestyle and also for early detection and appropriate interventions. Periodically educational courses on “smoking cessation” are suggested. More research is needed to identify moderators of long-term stressors on MetS in long distance drivers.

## Methods

During a health survey on long distance professional drivers to assess their occupational health state, drivers residing in West Azerbaijan province were screened for the presence of MetS. Randomly selected long distance professional divers aged 20–69 years were included in the study, using stratified sampling from December 2007 to March 2010. The main ethnic groups living in the West Azerbaijan province are Azeries (Turks) and Kurds. Those drivers who were working for less than one year and those who rejected to participate in the study were excluded. All participants signed written constant forms approved by the ethical committee of Urmia University of Medical Sciences.

### Medical history and clinical examination

According to a national protocol, each participant was interviewed by trained physicians and completed a questionnaire containing information on demographics, anthropometric profile, individual characteristics associated with the past medical history, and biochemical parameters. Waist circumference was measured at the level of the umbilicus in the standing position of subjects. After five minutes rest, the subjects' blood pressure was measured by Iranian Institute of Standards and Industrial Researches, using a standard mercury sphygmomanometer with a suitable cuff calibrated. Two consecutive diastolic and systolic blood pressures were recorded on the right arm. If the difference of the two-measurements exceeded 5% (i.e., >5 mmHg out of the 100 mmHg), blood pressure was measured for a third time. There were at least 30 seconds interval between these separate measurements, and the average of the two closest readings was considered for analyses.

The article "Prevalence of Metabolic Syndrome in Iranian Professional Drivers: Results from a Population Based Study of 12,138 Men" was published in 2012. Journal: PLoS One.

### Serum lipid and glucose analysis

Baseline blood samples were drawn into vacutainer tubes between 7:00 to 9:00 a.m. All the participants had fasted ≥10 h. Fasting plasma glucose and lipids were quantified at the time of specimen collection in the central laboratory of UMSU, a reference laboratory that has served Urmia residents for decades. Blood glucose and lipids, including triglycerides, and high-density lipoproteins were analyzed using a BT-3000 auto-analyzer (Biotecnica, Rome, Italy). The HDL cholesterol and triglyceride were assayed using enzymatic tests with commercially available kits (Pars Azmoon Inc., Iran). Plasma glucose was measured by the glucose-peroxidase colorimetric enzymatic method with a sensitivity of 5 mg/dL and intra-assay coefficients of variation (CV) 1.7% in lower limit and 1.4% in upper limit concentrations. Inter-assay CV for the assay was 1.1% in lower limit and 0.6% in upper limit concentrations. Fasting plasma glucose (FPG) more than 100 mg/dl was defined abnormal in this study. All samples were analyzed when daily internal quality control met the acceptable criteria.

### Definition of MetS

The IDF in 2005, has proposed a “consensus” definition of MetS in which waist circumference cut-off thresholds have been made based on ethnicity [32]. All subjects were screened for MetS using IDF criteria that included the presence of central adiposity on the basis of waist circumference ≥94 cm plus two or more of the following four factors: 1) elevated concentration of triglycerides(TG): ≥150 mg/dl (1.7 mmol/l); 2) reduced concentration of high-density lipoprotein cholesterol (HDL-C): <40 mg/dl (1.03 mmol/l); 3) elevated blood pressure: systolic blood pressure(SBP) ≥130 mmHg or diastolic blood pressure (DBP) ≥85 mmHg; and 4) elevated fasting plasma glucose(FBG) concentration ≥100 mg/dl (5.6 mmol/l). Normal weight was defined as BMI <25 kg/m2; overweight was defined as BMI ≥25 kg/m2; and obesity was defined as BMI ≥30 kg/m2.

The article "Prevalence of Metabolic Syndrome in Iranian Professional Drivers: Results from a Population Based Study of 12,138 Men" was published in 2012. Journal: PLoS One.

### Statistical analysis

Data are presented as frequencies, and percentages. STATA 8 software was used for data analysis. Continuous variables are expressed as mean ± standard deviation (SD). Pearson's chi-square test was applied to test the association of categorical variables, and ANOVA was used to compare the mean number of components of MetS among drivers of different age groups. A test for trend was used to compare the prevalence of MetS among age groups. Logistic regression analyses were used to explore the contribution of baseline variables as independent variables of MetS including: age, BMI, smoking habit, driving experiences and weekly duration of driving as a working in fixed sitting position. To be able to compare our results with that of other studies, the findings were standardized with the World Health Organization world standard population [33].
